This article has been retracted.

# Serum MMP-9 and SAA in the Diagnosis of Severe Pneumonia Caused by Radiotherapy of Esophageal Cancer

**DOI:** 10.1155/2021/6032546

**Published:** 2021-08-05

**Authors:** Yu Zhou, Li Liu, Wenjun Gu

**Affiliations:** ^1^Department of ICU, Zhuji People's Hospital, Shaoxing, Zhejiang Province 311800, China; ^2^Department of Pediatrics, Zhuji People's Hospital, Shaoxing, Zhejiang Province 311800, China; ^3^Department of Gastroenterology, The Ninth People's Hospital, Shanghai Jiaotong University School of Medicine, Shanghai 200011, China

## Abstract

**Objective:**

To explore the relationship and diagnostic value of serum MMP-9 and SAA in severe pneumonia (sCAP) caused by radiotherapy of esophageal cancer.

**Methods:**

A total of 144 esophageal cancer patients who underwent radiotherapy in our hospital from April 2016 to February 2018 were collected. Among them, 58 patients without radiation pneumonitis (RP) were in the control group, 49 patients with grade 1∼2 RP were in the radiation group, and 37 patients with sCAP were in the severe group. The levels of serum MMP-9 and SAA in every group of patients were detected. The ROC curve was used to determine the diagnostic value of serum MMP-9 and SAA in the diagnosis of RP and sCAP. The correlation between serum MMP-9 and SAA and the patient's lung function indexes was analyzed, and the logistic single-factor and multivariate analyses were performed to analyze the factors of sCAP in esophageal cancer radiotherapy.

**Results:**

PaO_2_, FVC, and FEV1 decreased in RP and sCAP, and PaCO_2_, white blood cells, serum MMP-9, and SAA levels increased (*P* < 0.05); serum MMP-9 and SAA were negatively correlated with lung function (*P* < 0.05); the AUC of serum MMP-9 and SAA in RP was 0.833 and 0.823, respectively, and the AUC of the two combined diagnosis of RP was 0.919. The AUC of serum MMP-9 and SAA in sCAP was 0.809 and 0.797, respectively, and the AUC of both combined diagnosis of sCAP was 0.873; logistics multivariate analysis found that serum MMP-9, serum SAA, double lung V5, and V20 were independent risk factors for sCAP caused by radiotherapy for esophageal cancer (*P* < 0.05).

**Conclusion:**

Serum MMP-9 and SAA increase in RP and sCAP and are negatively correlated with lung function in patients with pneumonia. They are independent risk factors for severe pneumonia caused by radiotherapy of esophageal cancer and have good diagnostic value.

## 1. Introduction

Esophageal cancer has a high morbidity and mortality rate in China, and it has always been the main malignant tumor that threatens the health of Chinese residents. The incidence rate ranks among the top 6 incidences of all malignant tumors and the top 4 mortality rates [1]. According to the physical status of patients with esophageal cancer, the pathological type of tumor, the scope of invasion, and the planned application of multiple treatment methods, including surgery, antitumor drugs, radiotherapy, and other methods, radiotherapy is one of the important treatment methods for esophageal cancer [2]. 70% of patients with esophageal cancer are in the middle-advanced stage at the time of treatment and have lost the opportunity of radical surgical resection, and more than 95% of the esophageal cancer pathological type is squamous cell carcinoma, which is relatively sensitive to radiation. The comprehensive treatment mode of radical radiotherapy can improve the middle-advanced stage survival of patients with esophageal cancer [3]. For the generalized application of radiotherapy, side effects have gradually appeared.

Radiation pneumonitis (RP) is an inflammatory response caused by damage to normal lung tissue in the radiation field after a variety of malignant tumors, including esophageal cancer, are damaged [4]. As the most common adverse reaction of chest radiotherapy, RP also limits the prescribed dose given by clinicians, which affects the treatment effect and patient prognosis. The incidence of RP is also high. According to statistics, some scholars have found that the risk of RP ≥ 2 grade after radiotherapy is about 22% in patients with esophageal cancer, while the risk of RP in elderly patients with esophageal cancer receiving radiotherapy can be as high as 52.4% [5]. This suggests that elderly patients with esophageal cancer need more attention when receiving radiotherapy. To avoid the occurrence of RP in clinic, a dose volume histogram (DVH) is often used to evaluate radiotherapy plans, among which mean lung dose (MLD) and V20 (receiving 20 Gy lung volume as a percentage of total lung volume) are often used as constraint indicators, but the effect is not good [6]. Moreover, there is no consensus on the current research on the application of DVH parameters to predict the occurrence of RP after radiotherapy. The occurrence of RP can cause symptoms such as cough, shortness of breath, and fever in the short term, and extensive fibrosis can occur in the long term, leading to lung function damage, respiratory failure, and seriously affecting the quality of life of patients. If it is allowed to develop, it will worsen to severe pneumonia (sCAP). sCAP is a common critical illness. Its clinical manifestations are mainly symptoms of persistent respiratory deterioration. The progress of the disease can lead to remodeling of the pulmonary vascular intima, continuous increase in left ventricular filling pressure, etc., and it has a high mortality rate [7,8]. Early detection and corresponding treatment is the key to sCAP treatment. However, there is a lack of reliable diagnosis and early predictors of the severity of pneumonia in clinical practice.

There are reports that matrix metalloproteinase 9 (MMP-9) and serum amyloid A (SAA) play a certain role in the process of sCAP [9]. Under normal circumstances, lung tissue only expresses a small amount of MMP-9, but under various stimuli, lung parenchymal cells such as bronchial epithelial alveolar cells, fibroblasts, smooth muscle cells, and endothelial cells can produce MMP-9. MMP-9 can degrade the extracellular matrix, increase the permeability of alveolar capillaries, promote the migration of multinucleated granulocytes, and promote inflammation. As a new indicator used to assist in the diagnosis of infectious diseases, SAA has received widespread attention in recent years. There is a certain correlation between the level of SAA and the severity of infection, and it has high specificity and sensitivity in diagnosing infection [10]. To this end, this study observed the serum levels of serum MMP-9 and SAA in patients with sCAP caused by radiotherapy for esophageal cancer, explored their diagnostic value in pneumonia, and analyzed the effects of the two and the physical factors of radiotherapy on the occurrence of sCAP, with a view to clinical practice providing reference for correct diagnosis and evaluation of RP and sCAP. The report is as follows.

## 2. Materials and Methods

### 2.1. Research Object

144 esophageal cancer patients undergoing radiotherapy were collected in our hospital from April 2016 to February 2018, including 91 males and 53 females, aged 51∼73 years, with an average age of 63.64 ± 10.6 years. Among them, 58 patients without radiation pneumonia were included in the control group, 36 were males and 22 were females, with an average age of 59.63 ± 11.7 years; 49 patients with grade 1-2 radiation pneumonia were included in the radiation group, 30 were males and 19 were females. With an average age of 60.25 ± 9.61 years; 37 patients with severe pneumonia belong to the severe group, with 25 males and 12 females, with an average age of 61.13 ± 12.41 years. There was no statistical difference between the three groups of general information (*P* > 0.05). All patients were given corresponding anti-infection, cough-relieving, and expectorant treatments according to their condition. This study did not require any intervention in the treatment of patients. The selected patients and their families were informed of the purpose, methods, and possible risks of the study and signed an informed consent form.

#### 2.1.1. Implementation Status of the Radiotherapy Plan

All patients received three-dimensional conformal radiotherapy, which was fixed by thermoforming, and localized CT scans with a thickness of 5 mm, including the middle and lower neck and the whole chest and upper abdomen. The images were transmitted to the Release 4.3.1 treatment system. The radiotherapy used a Varian23 EX. Linear Accelerator. The PTV of esophageal cancer was 5∼10 mm of CTV, the prescribed dose of radical radiotherapy was 60 Gy, and the prescribed dose of postoperative adjuvant radiotherapy was 50∼60 Gy, both of which shall be divided by 2 Gy/F routinely, with 98% isodose wire surrounding more than 95% of the planned target volume. Normal tissue limit: spinal cord dose < 45 Gy; heart V30 < 40%, V40 < 30%; average dose in both lungs < 20 Gy, V20 < 30%, V30 < 20%, and V20 limit in both lungs < 28% during concurrent chemotherapy. 144 patients with esophageal cancer received low-dose cisplatin/nedaplatin concurrent chemoradiation (44.5%).

#### 2.1.2. RP Diagnostic Criteria [11]

According to the patient's symptoms and signs such as cough, sputum, fever, and shortness of breath, in conjunction with physical examinations, chest X-rays, chest CT, and other examinations, the diagnosis is limited to the irradiation area, and the disease does not match the anatomical structure of normal lung tissue.

#### 2.1.3. sCAP Diagnostic Criteria

The diagnosis of sCAP refers to the diagnostic criteria of sCAP in the adult CAP diagnosis and treatment guidelines jointly promulgated by the American Society of Infectious Diseases and the American Thoracic Society in 2007: ①The main indicators include the need for forced mechanical ventilation, the appearance of septic shock, and the need for vasopressor drugs; ②secondary indicators, including respiratory rate 30 beats/min, PaO_2_/inhaled oxygen concentration (FiO_2_) ≤ 250, multiple-lobe infiltration, confusion or disorientation, uremia (blood urea nitrogen ≥ 7.14 mmol/L), leukopenia (white blood cells < 4.0 × 10^9^/L), thrombocytopenia (platelets < 100 × 10^9^/L), hypothermia (core body temperature < 36°C), and hypotension requiring active fluid resuscitation. It can be diagnosed as sCAP if it meets any one of the abovementioned main diagnostic criteria or any three of the secondary criteria.

#### 2.1.4. Exclusion Criteria

People with HIV infection, white blood cells <1 × 10^9^/L, or neutrophils <0.5 × 10^9^/L, those after organ transplantation use a glucocorticoid equal to or greater than 1 mg/(kg·d) prednisone, and those older than 1 month were not included in the study. Patients who died within 24 hours of enrollment and who withdrew halfway through were not included in the statistics.

### 2.2. Research Methods

#### 2.2.1. Clinical Data

Patient data (age, gender, etc.) were collected, and 5 ml of venous blood samples were collected on the day of admission or the morning after admission to the ICU. The content of white blood cells was detected, the arterial blood gas analysis (PaO_2_, PaCO_2_) was performed, and the patient's forced expiratory volume in 1-second (FEV1) and forced vital capacity (FVC) were detected by using a pulmonary function detector.

#### 2.2.2. Serum MMP-9 and SAA Levels

The level of serum MMP-9 was detected by enzyme-linked immunosorbent assay (ELISA), and the specific operation was carried out according to the manufacturer's instructions. The kit was purchased from Shanghai Ekosai Biological Products Co., Ltd., and the microplate reader was produced in Finland. Serum SAA levels were determined by using the specific protein analyzer P120 and supporting kits produced by Shenzhen Jinrui Company.

### 2.3. Statistical Methods

SPSS22.0 software was used for analysis, measurement data conforming to normal distribution were expressed as mean ± standard deviation, and a *t*-test was used for comparison between groups; correlation was detected by the Pearson correlation test; the differential diagnosis value of various indicators for radiation pneumonia and severe pneumonia was evaluated by the receiver operating characteristic (ROC) curve; the factors related to the occurrence of sCAP in serum MMP-9, SAA, and DVH parameters were analyzed by single-factor logistic regression; the statistically significant factors in the univariate analysis were included in the multivariate Logistic; and *P* < 0.05 indicated that the difference was statistically significant.

## 3. Results

### 3.1. Changes in Blood Routine and Lung Function of the Three Groups of Patients

The blood test results showed that compared with the control group, the radiation group and the severe group had lower PaO_2_, the PaCO_2_ and white blood cell increased, and the severe group had more obvious changes than the radiation group; pulmonary function tests showed that FVC and FEV1 of patients in the radiation group and the severe group were reduced, the severe group changed significantly compared with the radiation group, and the difference was statistically significant (*P* < 0.05), as shown in Figure 1.

### 3.2. Serum MMP-9 and SAA Levels of the Three Groups of Patients

Compared with the control group, the serum MMP-9 and SAA levels of patients in the radiation group and severe group increased, and the difference was statistically significant (*P* < 0.05); compared with the radiation group, the difference between serum MMP-9 and SAA in severely ill patients was not statistically significant (*P* > 0.05), as shown in Figure 2.

### 3.3. The Correlation between Serum MMP-9 and SAA and Lung Function

The Pearson correlation test showed that serum MMP-9 was strongly negatively correlated with FVC and FEV1 and serum SAA was weakly negatively correlated with FVC and FEV1, both of which were statistically significant (*P* < 0.05), as shown in Figure 3.

### 3.4. The Diagnostic Value of Serum MMP-9 and SAA for RP

The ROC curve showed that the area under the curve (AUC) of serum MMP-9 in RP was 0.833 and the AUC of serum SAA in RP was 0.823. The AUC of both combined diagnosis in RP was 0.919, both of which were statistically significant (*P* < 0.05), as shown in Table 1 and Figure 4.

### 3.5. The Diagnostic Value of Serum MMP-9 and SAA for sCAP

The ROC curve showed that the AUC of serum MMP-9 in sCAP was 0.809, the AUC of serum SAA in sCAP was 0.797, and the AUC of sCAP in the combined diagnosis of the two was 0.873, both of which were statistically significant (*P* < 0.05), as shown in Table 2 and Figure 5.

### 3.6. Factors Affecting sCAP Caused by Radiotherapy for Esophageal Cancer

Logistic single-factor analysis showed that serum MMP-9, serum SAA, lung V5 (*P* < 0.05), V10 (*P* < 0.05), V20 (*P* < 0.05), V30 (*P* < 0.05), and MLD (*P* < 0.05) all are related factors of sCAP caused by radiotherapy for esophageal cancer, and there are statistical differences (*P* < 0.05), as shown in Table 3; in the univariate analysis results, the DVH parameters that have a significant correlation with sCAP, serum MMP-9, serum SAA, double lung V5, V10, V20, V30, and MLD, were subjected to logistic multivariate analysis, the results showed that only the lung serum MMP-9 (*P* ≤ 0.001), SAA (*P* ≤ 0.001), V5 (*P*=0.017), and V20 (*P*=0.006) were statistically significant. It suggested that serum MMP-9, serum SAA, double lung V5, and V20 were independent risk factors for sCAP caused by radiotherapy for esophageal cancer; V10 (*P*=0.103) V30 (*P*=0.115) in both the lungs and MLD (*P*=0.437) were related to the occurrence of sCAP caused by radiotherapy for esophageal cancer, but they were not independent factors related to the occurrence of sCAP caused by radiotherapy for esophageal cancer, as shown in Table 4.

## 4. Discussion

RP, as one of the more common complications of radiotherapy for esophageal cancer, is the interaction of a variety of cells and molecules, which causes a large number of fibroblasts to accumulate, proliferate, and differentiate, cause excessive extracellular matrix deposition, and ultimately lead to pulmonary fibrosis and cause the pathology of the sCAP physiological process [12]. With the continuous update of radiotherapy technology and equipment, the efficacy of radiotherapy for esophageal cancer has improved. However, radiation-induced lung injury can occur in patients after radiotherapy, which can cause sCAP in severe cases, which significantly affects the patient's quality of life and prognosis and becomes an important factor limiting the increase in clinical radiotherapy dose [13]. Therefore, the research on radiation-induced lung injury has attracted more and more attention from scholars at home and abroad. However, the specific mechanism of the occurrence of RP and sCAP is still unclear, so traditional views still use MLD as the main factor in evaluating radiotherapy plans to reduce the risk of RP, but there is still no consensus. In clinical work, V20 < 30% MLD < 20∼23 Gy is used to avoid the occurrence of RP, but studies have shown that the effect is not good.

In recent years, the research on the mechanism of radiation-induced lung injury has mainly focused on cytokines. The cytokines closely related to the occurrence and development of radiation-induced lung injury mainly include transforming growth factor, plasma endothelin-1, tumor necrosis factor-*α*, etc. [14–16]. With the development of molecular biology, more reports believe that radiation-induced lung injury is mainly related to biological factors such as cytokines, and it is not a single cytokine function, but a complex and related interaction between multiple cytokines. Studies have shown that the MMP family has a certain mechanism of action in pneumonia and other diseases [17]. Among them, MMP-9 can degrade almost all extracellular matrix components such as collagen fibers, elastic fibers, and proteoglycans in the alveolar wall, induce the migration of polynuclear granulocytes, and change their morphology, thereby improving the permeability of microvessels and promoting the migration of polynuclear granulocytes., causing organ damage and the spread of inflammation, leading to systemic inflammatory response syndrome, and initiating the cascade of inflammatory response [18]. Pathological studies have shown [19] that the level of MMP-9 is basically the same as the degree of local lung inflammation and alveolar destruction under the microscope. SAA is a family of polymorphic proteins encoded by multiple genes, mainly derived from hepatocyte secretion, and is the precursor of tissue amyloid A. SAA levels are significantly increased in patients with bacterial and viral infections and can rise rapidly at the initial stage of infection and decline rapidly during the recovery period of the disease. The levels in children with bacterial and viral infections are significantly increased, especially in patients with bacterial infections. The most obvious increase is in children [20]. Studies have also shown [21] that SAA has a certain diagnostic value for bacterial pneumonia, but there are fewer studies on RP and sCAP.

The indicators such as MLD and double lung V20 in the radiotherapy plan have been widely used in clinical treatment plan evaluation. Since most studies mainly analyze the dose and volume parameters of the irradiated lung tissue from the perspective of radiation physics, it has certain guiding significance. However, due to the lack of organic integration with biology, the human body is a complex biological organism, so it is not completely correct to evaluate and predict the degree of radiation-induced lung injury. This study comprehensively analyzed the serum MMP-9 and SAA expression levels and the influence of physical factors in radiotherapy on RP and sCAP caused by radiotherapy for esophageal cancer and its diagnostic value. We first analyzed RP and sCAP blood routine and pulmonary function and other indicators. The results of the study showed that PaO_2_, FVC, and FEV1 decreased in RP and sCAP patients, PaCO_2_ and white blood cells increased, and the proportion of patients with a history of smoking was more, and the severe group was called the radiation group. The changes are obvious, suggesting that sCAP patients have more obvious index deterioration than RP patients, and attention should be paid to monitoring when RP occurs to reduce the production of sCAP as much as possible. Analysis of the levels of serum MMP-9 and SAA in patients showed that serum MMP-9 and SAA levels in patients with RP and sCAP were elevated. This may be related to the involvement of MMP-9 and SAA with inflammation and bacterial infection.

Analysis of the correlation between serum MMP-9 and SAA levels and lung function showed that serum MMP-9 was negatively correlated with FVC and FEV1 and serum SAA was negatively correlated with FVC and FEV1, suggesting that the two are negatively correlated with lung function. The ROC curve was used to predict the diagnostic value of serum MMP-9 and SAA levels for RP and sCAP. It was found that the AUC of serum MMP-9 and SAA in RP was 0.833 and 0.823. The AUC of the two combined diagnosis of RP was 0.919, the AUC of serum MMP-9 and SAA in sCAP was 0.809 and 0.797, and the AUC of the two combined diagnosis of sCAP is 0.873, indicating that the two have a good diagnostic value for RP and sCAP, and the diagnosis of RP is better than sCAP. Logistics multivariate analysis of serum MMP-9 and SAA levels and physical factors of radiotherapy found that serum MMP-9, serum SAA, double lung V5, and V20 are independent risk factors for sCAP caused by radiotherapy for esophageal cancer.

## 5. Conclusions

In summary, serum MMP-9 and SAA increase in RP and sCAP and are negatively correlated with lung function in patients with pneumonia. They are independent risk factors for severe pneumonia caused by radiotherapy for esophageal cancer and have good diagnostic value.

## Figures and Tables

**Figure 1:** Blood routine and lung function changes of the three groups of patients. Note: compared with the control group, ^*∗*^*P* < 0.05; compared with the radiation group, ^#^*P* < 0.05.

**Figure 2:** Serum MMP-9 and SAA levels of the three groups of patients. Note: compared with the control group, ^*∗*^*P* < 0.05.

**Figure 3:** Correlation between serum MMP-9 and SAA and lung function. Note: the *r* value represents the strength of the correlation.

**Figure 4:** ROC curve of serum MMP-9 and SAA for diagnosing RP.

**Figure 5:** ROC curve of serum MMP-9 and SAA in diagnosing sCAP.

**Table 1:** The diagnostic value of serum MMP-9 and SAA for RP.

Factor	AUC	S.E	95% CI	*P* value
Serum MMP-9	0.833	0.039	0.756∼0.910	<0.0001
Serum SAA	0.823	0.040	0.743∼0.902	<0.0001
Combined diagnosis	0.919	0.029	0.863∼0.975	<0.0001

**Table 2:** The diagnostic value of serum MMP-9 and SAA for sCAP.

Factor	AUC	S.E	95% CI	*P* value
Serum MMP-9	0.809	0.048	0.715∼0.904	<0.0001
Serum SAA	0.797	0.048	0.703∼0.891	<0.0001
Combined diagnosis	0.873	0.040	0.795∼0.951	<0.0001

**Table 3:** Logistic univariate analysis of severe pneumonia caused by radiotherapy for esophageal cancer.

Factor	*B*	df	Sig	Exp (*B*)	95% CI
Serum MMP-9 (*μ*g/L)	0.329	1	0.003	1.364	1.137∼1.964
Serum SAA (mg/L)	0.256	1	0.016	1.294	1.067∼1.648
V5 (%)	0.203	1	0.024	1.196	1.126∼1.296
V10 (%)	0.231	1	0.046	1.235	1.165∼1.207
V20 (%)	0.572	1	0.013	1.861	1.493∼2.064
V30 (%)	0.481	1	0.037	1.593	1.424∼1.872
MLD (Gy)	0.706	1	0.029	1.968	1.577∼2.393

**Table 4:** Logistic multivariate analysis of severe pneumonia caused by radiotherapy for esophageal cancer.

Factor	*B*	df	Sig	Exp (*B*)	95% CI
Serum MMP-9 (*μ*g/L)	0.031	1	≤0.001	1.031	1.017∼1.046
Serum SAA (mg/L)	0.248	1	≤0.001	1.281	1.155∼1.421
V5 (%)	0.123	1	0.017	1.133	1.026∼1.267
V10 (%)	0.010	1	0.103	1.009	0.873∼1.206
V20 (%)	0.401	1	0.006	1.457	1.126∼1.852
V30 (%)	0.173	1	0.115	1.182	0.967∼1.436
MLD (Gy)	−0.106	1	0.437	0.895	0.729∼1.162

## Data Availability

The data used and/or analyzed during the current study are available from the corresponding author.
